# Establishment and Evaluation of EGFR Mutation Prediction Model Based on Tumor Markers and CT Features in NSCLC

**DOI:** 10.1155/2022/8089750

**Published:** 2022-04-05

**Authors:** Hao Zhang, Meng He, Ren'an Wan, Liangming Zhu, Xiangpeng Chu

**Affiliations:** ^1^Department of Thoracic Surgery, Rizhao People's Hospital, Rizhao 276800, Shandong, China; ^2^Department of Thoracic Surgery, Jinan Central Hospital, Jinan 250013, Shandong, China

## Abstract

**Background:**

Lung cancer has become one of the leading causes of cancer deaths worldwide. EGFR gene mutation has been reported in up to 60% of Asian populations and is currently one of the main targets for genotype-targeted therapy for NSCLC.

**Objective:**

The objective is to determine if a complex model combining serum tumor makers and computed tomographic (CT) features can predict epidermal growth factor receptor (EGFR) mutation with higher accuracy. *Material and Methods*. Retrospective analysis of the data of patients diagnosed with in nonsmall cell lung cancer (NSCLC) by EGFR gene testing was carried out in the Department of Thoracic Surgery, Jinan Central Hospital. Multivariate logistic regression analysis was used to determine the independent predictors of EGFR mutations, and logistic regression prediction models were developed. The subject operating characteristic curve (ROC) was plotted, and the area under the curve (AUC) was calculated to assess the accuracy and clinical application of the EGFR mutation prediction model.

**Results:**

Logistic regression analysis identified the predictive factors of EGFR mutation including nonsmoking, high expression level of Carcinoembryonic Antigen (CEA), low expression level of cytokeratin 19 fragments (CYFRA21-1), and subsolid density containing ground-glass opacity (GGO) component. Using the results of multivariate logistic regression analysis, we built a statistically determined clinical prediction model. The AUC of the complex prediction model increased significantly from 0.735 to 0.813 (*p* *=* 0.014) when CT features are added and from 0.612 to 0.813 (*p* < 0.001) when serum variables are added. When *P* was 0.441, the sensitivity was 86.7% and the specificity was 65.8%.

**Conclusion:**

A complex model combining serum tumor makers and CT features is more accurate in predicting EGFR mutation status in NSCLC patients than using either serum variables or imaging features alone. Our finding for EGFR mutation is urgently needed and helpful in clinical practice.

## 1. Introduction

Lung cancer has become one of the leading causes of cancer deaths worldwide [1]. EGFR gene mutation has been reported in up to 60% of Asian populations and is currently one of the main targets for genotype-targeted therapy for NSCLC [2]. The discovery of structural domain activating mutations in EGFR tyrosine kinase promoted the concept of targeted therapy [3]. EGFR tyrosine kinase inhibitors (TKIs) were the first targeted agents for the treatment of NSCLC [4]. Currently, definitive diagnosis of EGFR mutation status is mainly detected from genomic DNA samples obtained from tumor tissues. However, tissue samples are difficult to obtain for EGFR mutation analysis, and tumor heterogeneity has an impact on accurate detection of EGFR mutations [5–7]. Circulating tumor DNA (ctDNA) in plasma samples can be an alternative method to detect EGFR mutations, but the results do not always agree with those of biopsy samples due to tumor heterogeneity, the false-negative rate is relatively high, and the cost is very high [4, 7, 8].

Serum tumor markers are mainly used in clinical practice to screen high-risk groups, observe and evaluate the effect of tumor treatment, and monitor the progression and recurrence of tumors. The results of the value of different serum tumor markers are inconsistent including significantly higher expression levels of CEA and carbohydrate antigen 199 (CA199), and lower expression level of CYFRA21-1 [4, 9–11].

In the diagnosis of lung cancer, CT is a routinely used and relatively cost-effective method that exhibits a variety of imaging features and can provide free data for genomics. Some studies have shown that the tumors typically presented with GGO were correlated with EGFR mutation [12, 13], while others found an inverse relationship or the lack of correlation [14]. In addition, other CT image features that have been found to be related with EGFR mutation include the maximum tumor diameter, spiculated margins, and the air bronchial sign [15, 16].

Although serum tumor markers and CT features show values in evaluating EGFR mutation status, the accuracy of these two methods by themselves is low. To our knowledge, it remains unclear whether the combination of these two methods can better diagnose EGFR mutation, and there are few studies combining these features to build predictive models. Therefore, we aim to construct a comprehensive model and evaluate its clinical application by analyzing serum tumor markers and CT imaging features in NSCLC patients.

## 2. Materials and Methods

### 2.1. Patient Selection

We included patients with pathologically diagnosed NSCLC between January 2018 and June 2020 at Jinan Central Hospital. Inclusion criteria included (1) pathological diagnosis of NSCLC by surgical resection, (2) serum tumor marker testing for lung cancer was performed at our hospital, (3) preoperative thin-section CT images, and (4) complete clinical information. Exclusion criteria included (1) no documented EGFR mutation testing, (2) history of previous antitumor therapy, (3) difficulty in outlining tumor margins, and (4) incomplete clinical data. Clinical data were collected, including patient gender, age, smoking history, pathological type, and clinical stage.

### 2.2. EGFR Mutation Detection

EGFR mutation was detected by experienced clinicians in the Department of Pathology of Jinan Central Hospital Hospital using surgically resected specimens. If an exon mutation was detected in EGFR exons 18–21, the tumor was considered to be EGFR mutant.

### 2.3. Measurement of Serum Tumor Maker Levels

The reference intervals for each index were CEA: 0–5 ng/ml, CYFRA21-1: 0–3.3 ng/ml, NSE: 0–16.3 ng/ml, CA125 : 0–35 U/ml, and CA199: 0–27 U/ml, respectively.

### 2.4. Image Acquisition and Feature Extraction

Images are viewed and analyzed by 2 imaging physicians in a double-blinded fashion on a PACS system. All examinations are extended in an intracranial direction with or without the use of contrast media. All images are archived in digital format. The following data were recorded: (1) maximum diameter (mm) of the lesion; (2) margins; (3) lesion density; and (4) lesion site. When 2 physicians disagreed, a higher level physician was asked to perform the analysis and reach a consensus result.

### 2.5. Statistical Analysis

The association of clinical characteristics, serum tumor marker levels, and CT image features with EGFR mutation was investigated by univariate analysis. The predictive factors of EGFR mutation was identified by logistic regression analysis and then built a statistically determined clinical prediction model. ROC was produced, and AUC was calculated to assess the accuracy of the prediction model. *p* < 0.05 was considered a statistically significant difference.

## 3. Results

### 3.1. Relationship between EGFR Mutation Status and Clinical Characteristics

A total of 148 NSCLC patients, 70 men (47.3%) and 78 women (52.7%), with a mean age of 62.9 ± 10.28 years, were included in this study. The patient EGFR mutation rate was 50.6%. The results showed that the mutation rate was significantly higher in women, in nonsmoking patients, and in adenocarcinoma patients, with statistically significant differences (*p* < 0.05), while the differences in age and clinical stage of tumors were not statistically significant (*p* > 0.05) when compared between the mutant and wild-type groups.

### 3.2. Correlation of EGFR Mutation with Serum Tumor Markers

The results showed that CYFRA21-1 levels were significantly higher in the wild-type group (*p* < 0.001); CA199 levels were higher in the mutant group, with statistically significant differences (*p* < 0.05), while CA125, CEA, and NSE levels in the mutant group were not statistically significant compared with those in the wild-type group (*p* > 0.05).

### 3.3. Correlation of EGFR Mutation with CT Features

The results showed that the maximum tumor diameter was larger in the wild-type group, and the difference was statistically significant (*p* < 0.05); the proportion of semisolid (with ground-glass density) was significantly higher in the mutant group (*p* < 0.001); and the differences in lesion location, lobulated sign, and spiculated margins were not statistically significant when compared between the mutant and wild-type groups (*p* > 0.05).

### 3.4. Possible Predictors and Prediction Model

Univariate logistic regression analysis identified independent predictors with statistical significance (Tables 1–3). Multifactorial analysis was performed using dichotomous logistic regression, and the results showed that nonsmoking (*p* = 0.003), high CA199 expression (*p* = 0.001), low expression of CYFRA21-1 (*p* < 0.001), and semisolid density containing GGO component (*P* = 0.003) were independent risk factors for the development of mutations in the EGFR gene (*p* < 0.05), as detailed in Table 4.

The clinical prediction model was established: *p* = e^x^/(1 + e^x^), *X* = −0.985 + (1.294 ∗ Smoking history) + (1.625 ∗ CA199) − (1.522 ∗ CYFRA21-1) + (1.602 ∗ Density), where smoking history was 1 (No) or 0 (Yes); CA199 and CYFRA21-1 was 1 (positive) or 0 (negative); and density was 1 (subsolid) or 0 (solid). The Hosmer–Lemeshow test was used for goodness of fit (*χ*^2^ = 7.530; *p* = 0.376), indicating a good fit of the model.

### 3.5. ROC to Assess Prediction Model Effectiveness

The area under the curve for serum tumor marker predictor and imaging index predictor ROC was 0.735 (95% CI: 0.654–0.817, *p* < 0.001) and 0.612 (95% CI: 0.521–0.703, *p* < 0.05), respectively. When serum tumor markers were combined with CT image features, the area under the curve of the integrated model was 0.813 (95% CI: 0.743–0.883, *p* < 0.001). The difference in AUC between the integrated model and the serum tumor marker predictors or imaging index predictors was statistically significant (*p* < 0.05). When the cut-off value was 0.441, the sensitivity Se was 86.7% and specificity SP was 65.8%, as shown in Figure 1.

## 4. Discussion

Although TKIs can improve the prognosis of patients with EGFR mutations and have significant efficacy in patients with gene mutations, the detection rate of EGFR mutation is lower than expected [17]. Biopsy, the gold standard for EGFR mutation detection, may be limited by the lack of available tissue samples because biopsy and cytology specimens are first used for histological testing to confirm cancer type. In addition, patient refusal to undergo invasive biopsy, location or size of the tumor, difficulty in biopsy sampling, and potential risk of cancer metastasis also limit detection rates [18]. In this study, we attempted to evaluate the effectiveness of a complex prediction model wherein serum markers and CT features are combined.

Previous demographic analyses have shown that a high prevalence of EGFR mutation is associated with female, nonsmokers, adenocarcinoma tissue type, and East Asian populations [4, 19], which is consistent with the our study results. Furthermore, we found that smoking history was an independent predictor of EGFR mutation by multivariate analysis, consistent with the study by Sabri et al. [20].

Serum tumor markers can be tested quickly and accurately in the hospital at a low cost [11]. Preoperative serum tumor markers have been shown to correlate with EGFR mutation and the efficacy of EGFR-TKI therapy [21]. Therefore, it is practical to use STMs to predict EGFR mutation [22]. Our current study demonstrated that the serum CA199 level was significantly higher in the EGFR mutation group while CYFRA21-1 was significantly increased in the wild-type group. Zhang et al. found that serum CEA levels could be used as a predictive tumor marker for the efficacy of EGFR-TKI therapy [23]. Our study did not identify a significant difference in the CEA levels, which is worth to note that over half (77 out of 148 cases) of our selected NSCLC patients were at an early stage of NSCLC development. The CA125 and NSE levels were not significantly altered by mutations in EGFR gene, consistent with a previous report [20].

CT is a routinely used and relatively economical modality for diagnosing lung cancer, and it presents a variety of imaging features that may be used to identify patients with NSCLC who are at risk for EGFR mutations. We found that EGFR mutation was associated with a smaller maximum diameter and subsolid density. Although univariate analysis found tumor size to be a factor associated with EGFR mutation, multifactorial analysis showed that tumor size was not a strong independent predictor, consistent with Rizzo et al. [24]. In addition, our study showed no significant differences in terms of lesion location, lobulated sign, and spiculated margins, which were consistent with some previous studies [20, 25] but contrary to the findings of Zhou et al. [26].

Although serum tumor markers and CT features can assess EGFR mutation status in NSCLC, the accuracy of predicting EGFR mutations by these two methods alone is not sufficient. To our knowledge, it remains unclear whether the combination of these two methods can better diagnose EGFR mutation status, and there are few clinical prediction models for EGFR mutations combining these features [20, 27]. We identified the independent predictors including nonsmoking, high CA199 expression, low CYFRA21-1 expression, and semisolid density containing a ground-glass opacity (GGO) component. The model was *p* = e^x^/(1 + e^x^), and *X* = -0.985 + (1.294∗Smoking history) + (1.625∗CA199) - (1.522∗CYFRA21-1) + (1.602∗Density). The AUC of the prediction model increased from 0.735 to 0.813 when CT feature predictors were added (*p* *=* 0.014) and from 0.612 to 0.813 when serum variables were added (*p* < 0.001). The cut-off point for 0.441 exhibited ideal sensitivity (86.7%) and acceptable specificity (65.8%).

## 5. Conclusion

In conclusion, EGFR mutation models constructed from serum tumor markers and CT features have good predictive efficacy. When properly combined, the complex model can have better predictive performance and higher diagnostic accuracy, facilitating clinical practice in identifying candidates for targeted therapy.

Our study has several limitations. First, it was a single-center retrospective study with a relatively small sample size and lack of external validation, which potentially compromise the generalization, sensitivity, and specificity of our model. Therefore, it needs to develop uniform standards for multicenter studies and to establish and test multicenter data. Second, squamous cell carcinoma (SCC) antigen was not included in this clinical prediction model due to incomplete documentation of these tumor markers in the HIS system. Therefore, we recommend refinement of our model prior to further validation. Finally, this study demonstrated that the integrated model has good predictive performance, but the accuracy is limited by its logistic regression method. Models built by different methods such as random forest and elastic network regression should be combined to develop the model.

## Figures and Tables

**Figure 1:** ROC curves for the complex model, serum predictors (CA199+CYFRA21-1), and imaging predictors (density) in differentiating EGFR mutation status.

**Table 1:** Relationship between clinical characteristics and EGFR mutation.

Characteristics	EGFR wild-type (*n* = 73)	EGFR mutations (*n* = 75)	*p*
Gender			<0.001
Female	25 (34.2%)	53 (70.7%)	
Male	48 (65.8%)	22 (29.3%)	
Age (years)	63.59 ± 10.47	60.63 ± 9.96	0.08
Smoking history			<0.001
Yes	40 (54.8%)	13 (17.3%)	
No	33 (45.2%)	62 (82.7%)	
Pathology type			0.037
AC	63 (86.3%)	72 (96.0%)	
Non-AC	10 (13.7%)	3 (4.0%)	
Clinical stage			0.101
I-II	33 (45.2%)	44 (58.7%)	
III-IV	40 (54.8%)	31 (41.3%)	

**Table 2:** Correlation of EGFR mutation with serum tumor markers.

Serum tumor markers	EGFR wild-type (*n* = 73)	EGFR mutations (*n* = 75)	*χ*2	*p*
CA125 (U/ml)			2.733	0.098
<35.0	52	62		
≥35.0	21	13		
CA199 (U/ml)			6.435	0.011
<27.0	57	44		
≥27.0	16	31		
CEA (ng/ml)			2.176	0.140
<5.0	39	49		
≥5.0	34	26		
NSE (ng/ml)			0.116	0.734
<16.3	60	60		
≥16.3	13	15		
CYFRA21-1 (ng/ml)			18.247	<0.001
<3.3	25	52		
≥3.3	48	23		

**Table 3:** Correlation of EGFR mutation with CT features.

CT features	EGFR wild-type (*n* = 73)	EGFR mutations (*n* = 75)	t/*χ*2	*p*
Maximum diameter (mm)	33.76 ± 20.85	26.83 ± 15.32	2.310	0.022
Density			10.689	0.001
Subsolid	8	25		
Solid	65	50		
Lesion location			3.080	0.079
Central	25	16		
Peripheral	48	59		
Lobulated sign			0.740	0.390
Yes	28	34		
No	45	41		
Spiculated margins			0.988	0.320
Yes	32	39		
No	41	36		

*Note.* Subsolid tumor contains GGO component.

**Table 4:** Result of multivariate logistic regression analysis.

Factors	B	S.E	Wals	*p*	OR	95%CI
Smoking history	1.294	0.430	9.042	0.003	3.649	1.569–8.483
CA199	1.625	0.473	11.799	0.001	5.077	2.009–12.829
CYFRA21-1	−1.522	0.432	12.417	<0.001	0.218	0.094–0.509
Density	1.602	0.547	8.595	0.003	4.964	1.701–14.488
Constant	−0.958	0.438	4.789	—	—	–

## Data Availability

The datasets used and/or analyzed during the current study are available from the corresponding author on reasonable request.
